RETRACTED

# LINC00092 Modulates Oxidative Stress and Glycolysis of Breast Cancer Cells via Pyruvate Carboxylase-Mediated AKT/mTOR Pathway

**DOI:** 10.1155/2022/5215748

**Published:** 2022-06-28

**Authors:** Wei Chen, Yushan Liu, Shaohong Kang, Xinying Lv, Wenfen Fu, Jie Zhang, Chuangui Song

**Affiliations:** ^1^Department of Breast Surgery, Fujian Medical University Union Hospital, Fuzhou, Fujian Province 350001, China; ^2^Department of General Surgery, Fujian Medical University Union Hospital, Fuzhou, Fujian Province 350001, China; ^3^Breast Cancer Institute, Fujian Medical University, Fuzhou, Fujian Province 350001, China

## Abstract

**Background:**

The discovery of noncoding RNAs (ncRNAs) offers new options for cancer-targeted therapy. This study is aimed at exploring the regulatory function of LINC00092 on breast cancer (BC) oxidative stress and glycolysis, along with internal mechanism concerning pyruvate carboxylase (PC).

**Methods:**

Bioinformatics analysis was used to explore LINC00092 (or friend leukemia virus integration 1 (FLI1)) expression on BC progression, as well as oxidative stress and glycolysis in BC. After LINC00092 overexpression or silence, BC cell viability, proliferation, migration, invasion, oxidative stress, glycolysis, and AKT/mTOR pathway were detected. Following 2-DG, SC79, or MK2206 treatment, effects of LINC00092 on BC cells were measured. Moreover, regulatory activity of LINC00092 in PC expression was analyzed. Whether PC participated in the modulation of LINC00092 on BC cell functions was explored.

**Results:**

LINC00092 was lowly expressed in BC and negatively related to BC progression. FLI1 bound to LINC00092 promoter to positively modulate LINC00092. LINC00092 overexpression inhibited BC cell proliferation, migration, invasion, oxidative stress, glycolysis, and AKT/mTOR pathway and likewise suppressed BC growth *in vivo*. Silence of LINC00092 had opposite influences. 2-DG partially reversed the LINC00092 silence-resulted increase of BC cell proliferation. SC79 alleviated the function of LINC00092 overexpression on BC cell functions. MK2206 had the contrary influence of SC79. Besides, LINC00092 bound to PC to modulate ubiquitination degradation of PC protein. PC took part in the influences of LINC00092 on BC cell functions.

**Conclusions:**

LINC0092 modulates oxidative stress and glycolysis of BC cells via the PC-mediated AKT/mTOR pathway, which is possibly a target for BC diagnosis and therapy.

## 1. Introduction

Breast cancer (BC) is the largest frequently happened cancer in women, which accounts for about 30% of all cancers happened in women [1]. Just in the United States, there are about 276,480 women diagnosed with BC in 2020 [2]. In recent years, with the development of targeted therapy and immunotherapy for BC, the overall prognosis of BC patients still remains discontented [3]. Cancer recrudescence and metastasis are two major causes for BC-related death [4]. It is well-known that the pathogenesis of BC is very complex. There are lots of molecules, in which expressions are changed in BC cells, due to gene mutation or chromosome variation [5–7]. Some of these are chosen to design targeted therapies for BC treatment [8, 9]. It is believed that more understanding of the pathogenesis of BC will provide new choices for exploring newly BC targeted therapy.

RETRACTED

Long noncoding RNAs (lncRNAs) are newly identified RNA transcripts with a length of more than 200 nucleotides in cells [10]. Different from well-known mRNAs, tRNAs, and rRNAs, which take part in encoding proteins, lncRNAs do not join in encoding proteins but exerted key regulatory roles in multiple cell functions [11]. More importantly, a number of lncRNAs are verified to bear a part in the tumorigenesis and progression of human cancers, including BC [12]. LINC00092 is firstly reported in 2017 and located at the intergenic regions of 9q22.32 [13]. Wang et al. [14] discovered that LINC00092 was lowly expressed in lung adenocarcinoma and predicated poor prognosis. Huang et al. [15] revealed that LINC00092 is a possible biomarker for colon adenocarcinoma diagnosis and prognosis. In terms of BC, Wu et al. [16] reported that LINC00092 expression was negatively correlated to the BC patients' survival outcomes.

Glycolysis refers to the process by which glucose is broken down into pyruvate in the cytoplasm under anaerobic condition [17]. For cancer cells, the proliferation is very quickly, which needs multiple adenosine triphosphate (ATP). Lots of literatures reported that glycolysis was promoted in many human cancer cells, including BC cells [18]. Actually, glycolysis is the main manner for BC cells to produce ATP, which is one of the important characteristics of malignant progression for BC [19, 20]. As key regulators of gene expressions in cells, many lncRNAs are discovered to take part in the modulation of glycolysis, including in BC cells [21, 22]. Chen et al. [23] found that LINC00092 could relieve cardiac fibroblast activation via regulating glycolysis. Zhao et al. [13] reported that LINC00092 could bind fructose-2,6-biphosphatase (PFKFB2) to modulate glycolysis in ovarian cancer cells. Not any information can be searched concerning the influence of LINC00092 on glycolysis of BC cells.

The redox imbalance, especially the increased level of oxidative stress, is demonstrated to happen in multiple human cancers, including BC [24]. Earlier literatures reported that raised oxidative stress not only took part in the BC formation via causing DNA and proteins damage but also participated in BC migration and invasion through altering expression changes of some molecules related to cell migration and invasion [25]. More importantly, it has been discovered that there is a reciprocal regulatory relationship between reactive oxygen species (ROS) and glycolysis in cells [26].

RETRACTED

In the current research, LINC00092 expression was detected in BC tissues to dissect the connection between LINC00092 expression and BC progression. The modulatory effect of friend leukemia virus integration 1 (FLI1) on LINC00092 expression in BC cells was analyzed. Following overexpression or silence of LINC00092 in BC cells, BC cell proliferation, migration, invasion, oxidative stress, glycolysis, and serine threonine (ser/thr) protein kinase/mammalian target of rapamycin (AKT/mTOR) pathway were tested. Moreover, whether LINC00092 influenced BC cell proliferation via regulating glycolysis and whether LINC00092 affected BC cell functions via AKT/mTOR pathway were analyzed. Finally, the internal regulatory mechanism of LINC00092 on BC cell metabolism concerning pyruvate carboxylase (PC) was probed. We think the findings of this research will provide experimental basis for further comprehending the key regulatory function of LINC00092 on BC progression.

## 2. Materials and Method

### 2.1. Bioinformatics Analysis

The RNA sequencing data of 1109 samples of BC tissues and 99 samples of normal tissues were downloaded from The Cancer Genome Atlas (TCGA) database (https://www.cancer.gov/about-nci/organization/ccg/research/structural-genomics/tcga) to dissect the connection among LINC00092 expression and BC progression. The RNA sequencing data of 1085 samples of BC tissues and 112 samples of normal tissues were downloaded from Gene Expression Profiling Interactive Analysis (http://gepia.cancer-pku.cn/) to dissect the connection among FLI1 expression and BC progression. Kaplan-Meier (KM) analysis was utilized to assess the influences of LINC00092 (or FLI1) expression on survival probability of BC patients. JASPAR website (https://jaspar.genereg.net/) was employed to explore the relationship between LINC00092 and FLI1. Gene Expression Profiling Interactive Analysis was also used to dissect the connection among FLI1 expression and LINC00092 expression in BC.

Gene Set Enrichment Analysis (GSEA, http://www.broad.mit.edu/gsea/msigdb/) was carried out to explore the enrichment of glycolysis and oxidative stress-related pathway modulated by LINC00092in BC tissues. Briefly, the clusterProfiler software package in an R package (http://bioconductor.org/packages/release/bioc/html/clusterProfiler.html.) was use in conducting gene ontology (GO) and Kyoto encyclopedia of genes and genomes (KEGG) enrichment analyses. Then, the GSEA of differentially expressed genes were analyzed using c2.cp.kegg.v6.2.symbols.gmt and c5.bp.v6.2.symbols.gmt in MsigDB V6.2 database (https://www.gsea-msigdb.org/gsea/msigdb/) as backgrounds. GESA was also performed using clusterProfiler package. Finally, the gene expressions concerning glycolysis and oxidative stress were analyzed using Bioinforcloud platform (http://www.bioinforcloud.org.cn).

RETRACTED

### 2.2. Clinical Samples

Twenty-nine BC patients were recruited in this research, which did not receive any therapy targeting BC before experiment. The BC tissues and paracancer normal tissues were harvested during surgical resection or pathological puncture biopsy. Written informed consents were obtained from patients. Experiments were authorized by the Ethics Committee of our institution.

### 2.3. Cell Culture

MCF-10A, MCF-7, MDA-MB-468, and MDA-MB-453 were cultured in corresponding medium recommended by the manufacturer at 37°C with 5% CO_2_. 5 mM 2-deoxyglucose (2-DG, D8930, Solarbio, Beijing, China) was used to inhibit cell glycolysis. 3 *μ*M SC79 (SF2730, Beyotime Biotechnology, Shanghai, China) was used to activate AKT, while 3 *μ*M MK2206 (SF2712, Beyotime Biotechnology) was used to inhibit AKT. 50 *μ*g/mL cycloheximide (CHX, HY-12320, MCE) was utilized to inhibit protein synthesis in cells.

### 2.4. Quantitative Polymerase Chain Reaction (qPCR) Assay

Total RNAs were separated from tissues or cells using Trizol solution (Invitrogen, CA, USA) and quantified via a microspectrophotometer (Hangzhou Allsheng Instruments Co., Ltd. Hangzhou, China). PrimeScript™ RT Reagent Kit with gDNA Eraser (Takara Biotechnology, Beijing, China) was utilized to synthesize cDNA with 2 *μ*g RNA as template. PCR assay was performed using SYBR Green qPCR Mix (Beyotime Biotechnology, Shanghai, China). Primer's sequences are exhibited in Table 1. Results were computed via the 2^-△△Ct^ method with GAPDH as endogenous control.

### 2.5. Cell Transfection

FLI1, LINC00092, and PC overexpression plasmids were erected via inserting the full-length sequences of FLI1, LINC00092, and PC into the pcDH plasmid (GeneChem Corporation, Shanghai, China), respectively. pLKO short hairpin RNA (shRNA) plasmids targeting LINC00092 and PC were designed to silence LINC00092 and PC expressions, which were synthesized by GeneChem Corporation and referred as sh-LINC00092 and sh-PC, respectively. sh-LINC00092 sequence was 5′-CCGGGGATGACCTGCCCTATGATTTCTCGAGAAATCATAGGGCAGGTCATCCTTTTTGAATT-3′. sh-PC sequence was 5′-CCGGCGACTCTGTGAAACTCGCTAACTCGAGTTAGCGAGTTTCACAGAGTCGTTTTTGAATT-3′. Cell transfection was carried out using Lipo8000™ Transfection Reagent (Beyotime Biotechnology, Shanghai, China).

RETRACTED

### 2.6. Chromatin Immunoprecipitation (ChIP) Assay

ChIP assay was utilized to dissect the connection of LINC00092 and FLI1 with the help of ChIP Assay Kit (Beyotime Biotechnology) [27]. FLI1 antibody was purchased from Invitrogen (MA1-196). DNA purification kit (AxGen, CA, USA) was used for DNA purification. qPCR was carried out for test LINC00092 expression. The LINC00092 primer sequences for ChIP were 5′-CAGATGCTCAGTGTGTGACCCT-3′ (forward) and 5′-CTGGGAACGGATGCGACAGT-3′ (reverse).

### 2.7. Dual-Luciferase Activity Assay

Dual-luciferase activity assay was utilized to further dissect the connection of FLI1 and LINC00092 with the help of Firefly and Renilla Luciferase Reporter Assay Kit (MeilunBio, Dalian, China) [28]. Briefly, MCF-7 and MDA-MB-468 cells were cotransfected into FLI1 and pGL3-LINC00092-WT (or pGL3-LINC00092-MUT, the 5′-TCAGGAAGCGC-3′ sequence of LINC00092 wild type was mutated with 5′-GTGTTGGTTTT-3′). After 48 h, total proteins in cells were separated. 20 *μ*L cell lysis supernatant was incubated with 100 *μ*L Firefly luciferase reaction buffer and 100 *μ*L Renilla detection kit. The relative luciferase activity was tested through a microplate reader.

### 2.8. Cell Counting Kit-8 (CCK-8) Assay

After corresponding transfection and/or treatment, 1 × 10^4^ cells were grown into a 96-well plate for 24, 48, and 72 h. Then, 10 *μ*L CCK-8 solution (Beyotime Biotechnology) was replenished into culture medium for 1 h [29]. Following shaking, the absorbance of each well was gauged at 450 nm.

### 2.9. Colony Formation Assay

After corresponding transfection and/or treatment, cells were cultivated into a 6-well plate with 500 cells/well for two weeks. Then, cells were rinsed by PBS, fixed with 4% paraformaldehyde solution (Beyotime Biotechnology), and dyed using Giemsa solution (Solarbio, Beijing, China). The colony number of each group was counted under a microscope.

### 2.10. Cell Scratch Assay

After corresponding transfection and/or treatment, 5 × 10^5^ cells were cultivated into a 6-well plate overnight. Then, scratches were generated by 10 *μ*L pipette across cells [30]. PBS was used to remove scratched cells. Following growth in culture medium that does not contain FBS at 37°C for 24 h, images of scratches were photographed under a microscope. The scratch areas were calculated using IPP software. The percentage of wound closure was calculated via 1 − (scratch area of 24 h/scratch area of 0 h × 100%).

### 2.11. Two-Chamber Transwell Assay

After corresponding transfection and/or treatment, 3 × 10^4^ cells in 200 *μ*L FBS-free culture medium were added into the above chamber that was pretreated with Matrigel Basement Membrane Matrix (Corning Costar, MA, USA) for 48 h [31]. 500 *μ*L culture medium containing 10% FBS was supplemented into the below chamber. Then, cells in the above chamber were removed and cells in membrane were cleaned using PBS, fixed with 4% paraformaldehyde solution, and dyed using 0.1% crystal violet solution. Results were photographed under a microscope.

RETRACTED

### 2.12. Animal Experiment

Twelve BALB/c nude mice (4 weeks old, female) were housed in aseptic environment at 26-28°C for 1 week to adopt to a new environment. Then, mice were weighted and randomly divided into the mock group and LINC00092 group. In mock group, mice were subcutaneously inoculated into the upper back area of right side with 1 × 10^6^ MDA-MB-468 cells transfected pcDH plasmid. In LINC00092 group, mice were subcutaneously inoculated with 1 × 10^6^ cells transfected LINC00092 plasmid. Body weight and tumor volume were measured at day 3, day 7, day 14, day 21, and day 28 (twice one week). After 28 days, all mice were sacrificed by CO_2_ inhalation. Tumor tissues were excised from mice, weighted, and fixed into 10% formalin solution. Hematoxylin-eosin staining was carried out to inspect the microstructure changes of tumor tissues between the mock and LINC00092 groups by using hematoxylin solution (G1004, Servicebio, Wuhan, China) and eosin solution (G1002, Servicebio).

## 3. Detection of Cell Glycolysis

Lactate production and glucose consumption of cells were tested with the help of lactate assay kit (A019-2-1) and glucose assay kit (F006-1-1, Nanjing Jiancheng Bioengineering Institute, Nanjing, China), respectively.

### 3.1. Test of Superoxide Dismutase (SOD) and Malondialdehyde (MDA) Level

SOD and MDA levels in MCF-7 and MDA-MB-468 cells after LINC00092 or sh-LINC00092 transfection were detected with the help of SOD Activity Detection Kit (BC0175, Solarbio) and MDA Detection Kit (S0131M, Beyotime Biotechnology) [32].

### 3.2. Measurement of ROS Level

ROS levels in cells were measured via ROS Assay Kit (S0033M, Beyotime Biotechnology) [33]. Briefly, after LINC00092 or sh-LINC00092 transfection, MCF-7 and MDA-MB-468 cells were rinsed with PBS and incubated with 10 *μ*mol/L DCFH-DA for 20 min at 37°C. Following rinsing with serum-free culture medium, the ROS levels in cells were tested via a microplate (488 nm excitation and 525 nm emission).

### 3.3. RNA Pull-Down and Mass Spectrometry (MS) Assay

RNA pull-down assay and MS analysis were performed to identify proteins interacting with LINC00092 [34]. Briefly, 1 × 10^7^ MDA-MB-468 cells were mixed with RIP Lysis Buffer on ice. Following centrifugation with 13000 × g for 10 min, supernatant was collected. LINC00092 *in vitro* transcription and purification were carried out using PrimeSTAR Max Premix (Takara Biotechnology, Beijing, China) and Micro-Agarose gel DNA recovery kit (Aiji Biotechnology, Guangzhou, China). mMESSAGE mMACHINE Kit (Invitrogen) and RNeasy Mini Kit were used to label LINC00092 with biotin. 3 *μ*g LINC00092 with biotin labeling was mixed with beads for 1 h. Cell supernatant was incubated with LINC00092-bead for 1 h. The LINC00092 binding proteins were eluted and collected to perform western blotting. MS analysis was performed using Thermo Scientific Q Exactive (ThermoFisher Scientific, MA, USA) with Proteome Discoverer 1.4 (version 1.4.0.288).

RETRACTED

### 3.4. RNA Immunoprecipitation (RIP) Assay

RIP was employed to further verify the binding of LINC00092 and PC. Magna RIP RNA-Binding Protein Immunoprecipitation Kit was purchased from Merck (#17-700, MA, USA), which was utilized in the light of the manufacturer's instruction. Results were tested by qPCR.

### 3.5. RNA-FISH Assay

RNA-FISH assay was performed to test the location of LINC00092 and PC in cells with the help of RNA-FISH Probe kit (Streptavidin-biotin system, GenePharma Biotechnology, Shanghai, China) [35]. LINC00092 probe sequence was 5′-CCAAATCATAGGGCAGGTCATCCCAAGGACAGCA-3′. PC probe sequence was 5′-GCAGTGAAGTCCTTGAAGTGGGCAAACACATCGGG-3′. DAPI (Solarbio) was utilized for staining nucleus.

### 3.6. Immunohistochemistry (IHC) Assay

Tumor tissues of mice were embedded using paraffin. Immunohistochemistry assay was performed on 6 *μ*m thick sections as earlier literature reported [36]. Anti-PC polyclonal antibody (#16588-1-AP), anti-Ki-67 polyclonal antibody (#21309-1-AP, Proteintech, IL, USA), anti-AKT (phospho T308) antibody (ab38449), anti-mTOR (phospho S2448) antibody (ab109268, Abcam Biotechnology, CA, USA), and anti-phosphor-p70 S6 kinase (Thr389) antibody (#97596) were purchased from Cell Signaling Technology, CA, USA. Relative expressions were visualized using diaminobenzidine (DAB) solution (Beyotime Biotechnology). Cell nucleus was stained using hematoxylin solution. Results were observed under a microscope (Nikon, Japan).

### 3.7. In Vitro Ubiquitination Assay

*In vitro* ubiquitination assay was carried out to identify the degradation pathway of PC protein modulated by LINC00092 in BC cells. Briefly, following different transfections, MCF-7 and MDA-MB-468 cells were treated by 20 *μ*M MG132 for 10 h (S1748, Beyotime) to inhibit degradation of ubiquitinated proteins [37]. RIPA Lysis Buffer (Beyotime Biotechnology) was used to split cells. The lysate supernatant was collected for co-immunoprecipitation with anti-IgG antibody or anti-PC antibody (#16588-1-AP, Proteintech). After incubation with Protein A/G Agarose and centrifugation and precipitation with Protein A/G Agarose, the protein in supernatant was subjected to western blotting.

RETRACTED

### 3.8. Western Blotting

Total proteins in cells were isolated using RIPA Lysis Buffer containing protease inhibitors and phosphatase inhibitors. Western blotting was conducted similarly as previous literature reported [38]. Anti-AKT antibody (ab8805), anti-p-AKT antibody (ab38449), anti-mTOR antibody (ab32028), and anti-p-mTOR antibody (ab109268) were purchased from Abcam Biotechnology. Anti-p70S6K antibody (#9202) and anti-p-p70S6K antibody (#97596) were provided by Cell Signaling Technology. Anti-PC antibody (#16588-1-AP) was purchased from Proteintech. Anti-GAPDH antibody (GB11002) was purchased from Servicebio.

### 3.9. Statistical Analysis

GraphPad Prism 9.0 software was utilized for statistical analysis. All experiments were repeated at least three times (*n* ≥ 3). Results were exhibited as mean ± standard deviation (SD). One-way ANOVA was utilized for gauging *P* values with a significance level of *P* < 0.05.

## 4. Results

### 4.1. LINC00092 Was Lowly Expressed in BC and Negatively Related to BC Progression

Firstly, the RNA sequencing data of BC tissues (T group) and normal tissues (N group) were downloaded from TCGA database to test LINC00092 expression. Result in Supplemental Figure 1A showed that relative to normal tissues, LINC00092 was lowly expressed in BC tissues (*P* < 0.0001). The BC tissues and paracancer normal tissues of 29 cases of BC patients were also collected. Supplemental Figure 1B also displays that LINC00092 had a lower expression level in BC tissues (*P* = 0.0001). Moreover, Supplemental Figure 1C illustrates that LINC00092 had lower expression levels in BC MCF-7 and MDA-MB-468 cells, in comparison with normal breast epithelial MCF-10A cells (*P* < 0.01). Besides, the relationship of LINC00092 expression and the tumor size, histological grade, and survival probability of BC patients was analyzed. Results showed that LINC00092 expression was negatively correlated with the tumor size (Supplemental Figure 1D, *P* = 0.01) and histological grade (Supplemental Figure 1E, Phase II and Phase III, *P* = 0.04) of BC patients. Supplemental Figure 1F displays that LINC00092 expression was positively related to the survival probability of BC patients (*P* < 0.0001). These outcomes represented that LINC00092 was lowly expressed in breast cancer tissues and cells and negatively associated with the BC progression.

RETRACTED

### 4.2. LINC00092 Was Modulated by FLI1 in BC Cells

Bioinformatics analysis found that there were complementary paired bases between the FLI1 motif and the LINC00092 promoter (Figure 1(a)).  Figure 1(b) shows that LINC00092 expression was positively related to FLI1 expression in BC (*P* = 4.1*E* − 55). Moreover, Figure 1(c) displays that FLI1 transfection notably raised the FLI1 expression in MCF-7 and MDA-MB-468 cells (*P* < 0.001), which also notably enhanced the LINC00092 expression in cells (Figure 1(d), *P* < 0.05 or *P* < 0.001). The results of ChIP in Figures 1(e) and 1(f) illustrated that FLI1 could be combined with LINC00092 promoter in cells (*P* < 0.001). Furthermore, the results of dual luciferase activity assay presented that cotransfection with LINC00092-WT and FLI1 notably raised the relative luciferase activities (Figures 1(g) and 1(h), *P* < 0.001). Besides, bioinformatics analysis also found that FLI1 was lowly expressed in BC tissues (Supplemental Figure 2A, 2*P*<0.05). BC patients with lower FLI1 expression had lower survival probability (Supplemental Figure 2B, *P* = 0.022). These outcomes represented that FLI1 bound to LINC00092 promoter to modulate LINC00092 expression in BC cells.

### 4.3. LINC00092 Regulated BC Cell Proliferation, Migration, and Invasion

LINC00092 and sh-LINC00092 were transfected to alter LINC00092 expression in MCF-7 and MDA-MB-468 cells.  Figure 2(a) displays that LINC00092 transfection raised the LINC00092 expression in cells (*P* < 0.001), while sh-LINC00092 transfection had opposite influence, which lowered LINC00092 expression in cells (*P* < 0.001).  Figure 2(b) shows that LINC00092 transfection reduced cell viabilities (*P* < 0.05 or *P* < 0.001), but sh-LINC00092 transfection enhanced cell viabilities (*P* < 0.01 or *P* < 0.001). Moreover, LINC00092 transfection inhibited cell proliferation (Figure 2(c)). Relative to the mock group, the number of foci/well was decreased in the LINC00092 group (*P* < 0.05 or *P* < 0.001). sh-LINC00092 transfection had contrary effect, which promoted cell proliferation (*P* < 0.01). Moreover, Figure 2(d) illustrated that LINC00092 transfection inhibited the cell migration (*P* < 0.01 or *P* < 0.001), but sh-LINC00092 transfection accelerated cell migration (*P* < 0.05). Besides, Figure 2(e) showed that LINC00092 transfection also reduced cell invasion (*P* < 0.01 or *P* < 0.001). sh-LINC00092 transfection had opposite effects, which facilitated cell invasion (*P* < 0.01 or *P* < 0.001). These outcomes represented that LINC00092 participated in the regulation of BC cell proliferation, migration, and invasion.

### 4.4. LINC00092 Overexpression Inhibited BC Growth In Vivo

An *in vivo* BC mouse model was established with MDA-MB-468 cells transfected or nontransfected LINC00092. Results in Figure 3(a) displayed that there was no notable difference of mouse body weight among the mock and LINC00092 group (*P* > 0.05).  Figure 3(b) presents that LINC00092 transfection inhibited the tumor volume of mice with BC (*P* < 0.001). The visual picture of mice with subcutaneous BC transplantation is shown in Figure 3(c).  Figure 3(d) shows that LINC00092 transfection also reduced the tumor weight of mice with BC (*P* < 0.001). Results of HE staining in Figure 3(e) showed that the compact tumor cells with blue-purple nuclei and pink cytoplasm were observed in the mock group. In the LINC00092 group, the tumor cells were separated each other with apparent vacant sections. Besides, relative to the mock group, the Ki-67 expression was decreased in the LINC00092 group, which further suggested that LINC00092 suppressed BC cell proliferation. These outcomes represented that LINC00092 overexpression inhibited BC growth *in vivo*.

RETRACTED

### 4.5. LINC00092 Influenced BC Cell Oxidative Response and Glycolysis

Both glycolysis and oxidative stress are demonstrated to be activated in BC tissues [20, 25]. Herein, the result of GSEA implied that both glycolysis and response to oxidative stress were regulated by LINC00092 in BC tissues (Figure 4(a)). Following LINC00092 or sh-LINC00092 transfection, cell relative lactate production and glucose consumption were measured. Figures 4(b) and 4(c) show that LINC00092 transfection reduced cell lactate production and glucose consumption (*P* < 0.05 or *P* < 0.01), while sh-LINC00092 transfection enhanced the lactate production and glucose consumption (*P* < 0.05, *P* < 0.01, or *P* < 0.001). 2-DG was utilized to inhibit glycolysis. Figures 4(d) and 4(e) display that 2-DG treatment reduced cell viabilities and colony formation (*P* < 0.05, *P* < 0.01, or *P* < 0.001). Moreover, the 2-DG combined with sh-LINC00092 significantly inhibited cell viabilities and colony formation compared with shLINC00092 alone (*P* < 0.01 or *P* < 0.001). Besides, Figure 4(f) shows that LINC00092 transfection raised the SOD level but lowered the MDA and ROS levels in MCF-7 and MDA-MB-468 cells (*P* < 0.001), while sh-LINC00092 transfection had opposite effects (*P* < 0.001). These outcomes represented that LINC00092 influenced BC cell glycolysis and oxidative response.

### 4.6. LINC00092 Influenced BC Cell Functions and Glycolysis via Modulating the AKT/mTOR Pathway

The AKT/mTOR pathway is a key proproliferation pathway in cells, which participates in the modulation of cell proliferation, migration, invasion, and glycolysis [39]. Whether AKT/mTOR pathway took part in the regulation of LINC00092 on BC cells was analyzed.  Figure 5(a) shows that LINC00092 inactivated the AKT/mTOR pathway in MCF-7 and MDA-MB-468 cells via reducing p-AKT, p-mTOR, and p-p70S6K protein levels. sh-LINC00092 transfection had contrary influence, which activated the AKT/mTOR pathway.  Figure 5(b) displays that LINC00092 also lowered the p-mTOR and p-p70S6K expressions in mouse xenograft BC tissue. SC79 was an activator of AKT, which reversed the inactivation of the AKT/mTOR pathway caused by LINC00092 transfection in cells (Supplemental Figure 3A). Figures 5(c)–5(f) display that SC79 treatment notably alleviated the LINC00092 transfection-resulted decreases of cell viabilities, proliferation, migration, and invasion (*P* < 0.05, *P* < 0.01, or *P* < 0.001). Furthermore, SC79 treatment also obviously relieved the LINC00092 transfection-resulted reductions of cell lactate production and glucose consumption (Figures 5(g) and 5(h), *P* < 0.01 or *P* < 0.001). MK2206 was an inhibitor of AKT. The results in Supplemental Figures 3B–3H illustrated that MK2206 treatment reversed the sh-LINC00092 transfection-resulted AKT/mTOR activation, cell viabilities, proliferation, migration, and invasion enhancements, as well as increases of lactate production and glucose consumption (*P* < 0.01 or *P* < 0.001). These outcomes represented that LINC00092 influenced BC cell viability, proliferation, migration, invasion, and glycolysis which could be via modulating the AKT/mTOR pathway.

RETRACTED

### 4.7. LINC00092 Regulated Ubiquitination Degradation of PC Protein in BC Cells

RNA pull-down assay and MS analysis were carried out to identify proteins interacting with LINC00092 in BC cells. Figures 6(a) and 6(b) illustrate that LINC00092 could bind to PC protein. The results of RNA-FISH assay in Figure 6(c) display that LINC00092 colocalized with PC protein in the cytoplasm of MCF-7 and MDA-MB-468 cells. The results of western blotting following RNA pull-down displayed that LINC00092 bound with PC (Figure 6(d)). Similar results were found in RIP assay in Figure 6(e). Relative to the IgG group, the relative enrichments of PC protein in the anti-PC group were significantly increased in cells (*P* < 0.001). These outcomes suggested that LINC00092 interacted with PC in BC cells. Next, the molecular mechanism of the interaction between LINC00092 and PC was explored. Results showed that LINC00092 or sh-LINC00092 transfection had no significant effect on PC mRNA expression (Figure 6(f), ^n.s.^*P* > 0.05) but negatively regulated PC protein level in cells (Figure 6(g)). LINC00092 transfection notably lowered the PC protein expression in cells (*P* < 0.05 or *P* < 0.001), while sh-LINC00092 transfection obviously raised the PC protein expression in cells (*P* < 0.05 or *P* < 0.001). The results of immunohistochemistry assay in Figure 6(h) further displayed that LINC00092 transfection reduced the PC protein expression in mouse xenograft BC tissue. Therefore, we speculated that LINC00092 might regulate the protein stability of PC in BC cells. CHX was used to inhibit protein (including PC) synthesis in cells. The results in Figure 6(i) showed that LINC00092 transfection promoted the degradation of PC protein (*P* < 0.05 or *P* < 0.01), while sh-LINC00092 transfection inhibited the degradation of PC protein in cells (*P* < 0.05 or *P* < 0.01). The protein degradation mediated by the ubiquitin proteasome pathway is the main mechanism for the body to regulate intracellular protein levels, which participates in the degradation of more than 80% of intracellular protein [40]. The results of *in vitro* ubiquitination assay in Figure 6(j) displayed that LINC00092 modulated the degradation of PC protein in BC cells via the ubiquitination pathway. These above outcomes represented that LINC00092 regulated ubiquitination degradation of PC protein in BC cells.

RETRACTED

### 4.8. PC Participated in the Regulation of LINC00092 on BC Cell Functions

PC was transfected to raise PC level in cells.  Figure 7(a) illustrates that compared to the LINC00092 group, the PC protein level in the LINC00092+PC group was increased in cells (*P* < 0.05 or *P* < 0.01). Following LINC00092 and/or PC transfection, cell viabilities, proliferation, migration, invasion, and glycolysis were detected. Results in Figures 7(b)–7(e) showed that PC transfection promoted cell viabilities, proliferation, migration, and invasion (*P* < 0.01 or *P* < 0.001). Relative to the LINC00092 group, cell viabilities, proliferation, migration, and invasion in the LINC00092+PC group were decreased (*P* < 0.05, *P* < 0.01, or *P* < 0.001), which presented that PC transfection weakened the influence of LINC00092 transfection on cell viabilities, proliferation, migration, and invasion. Similar results were found for the glycolysis of MCF-7 and MDA-MB-468 cells. Figures 7(f) and 7(g) illustrate that PC transfection elevated the cell lactate production and glucose consumption (*P* < 0.01 or *P* < 0.001), as well as alleviated the LINC00092 transfection-resulted reductions of lactate production and glucose consumption (*P* < 0.05 or *P* < 0.01). Besides, sh-PC was transfected to silence PC expression in cells. Results in Supplemental Figures 4A–4G showed that silence of PC partially reversed the influences of sh-LINC0092 transfection MCF-7 and MDA-MB-468 cell viabilities, proliferation, migration, invasion, and glycolysis (*P* < 0.05, *P* < 0.01, or *P* < 0.001). These above outcomes represented that overexpression of PC weakened the influences of LINC00092 transfection on BC cell functions.

RETRACTED

### 4.9. PC Participated in the Modulation of LINC00092 on the AKT/mTOR Pathway in BC Cells

Finally, following PC and/or LINC00092 transfection (or sh-PC and/or sh-LINC00092 transfection), the activity of the AKT/mTOR pathway in cells was measured. Results displayed that PC transfection activated the AKT/mTOR pathway in cells by enhancing p-AKT/AKT, p-mTOR/mTOR, and p-p70S6K/70S6K protein levels (Supplemental Figure 5A, *P* < 0.01 or *P* < 0.001), as well as reversed the LINC00092 transfection-resulted inactivation of the AKT/mTOR pathway (*P* < 0.05, *P* < 0.01, or *P* < 0.001). Besides, sh-PC had opposite influence, which inactivated the AKT/mTOR pathway in cells by lowering p-AKT/AKT, p-mTOR/mTOR, and p-p70S6K/70S6K protein levels (Supplemental Figure 5B, *P* < 0.01 or *P* < 0.001), as well as weakened the sh-LINC00092 transfection-resulted activation of the AKT/mTOR pathway (*P* < 0.05 or *P* < 0.01). These outcomes suggested that PC play a key role in the modulation of LINC00092 on the AKT/mTOR pathway in BC cells.

## 5. Discussion

As the most common malignant cancer in women, BC threats the health and life of many individuals, which also brings great mental and financial pressures for BC patients [2, 41]. In recent years, lncRNAs are verified to serve as a key regulator of gene expression in eukaryotic cells [42]. More importantly, lots of lncRNAs are discovered to take part in the progression of human cancers, which offers a new direction for cancer-targeted therapy [11]. There are many clinical trials concerning the roles of lncRNAs in cancer diagnosis and therapy, which can be inquired in Clinicaltrials.gov database (https://clinicaltrials.gov). LINC00092 was a newly discovered lncRNA. Wu et al. [16] reported that LINC00092 expression was significantly associated with the survival of BC patients. Zhao *et al.* [43] discovered that LINC00092 expression was downregulated in breast invasive ductal carcinoma (BIDC) tissues and cells, which promoted malignant progression of BIDC via regulating secreted frizzled related protein 1 (SFRP1) by sponging microRNA-1827. Herein, we revealed that LINC00092 had lower expression level in BC tissues and cells and negatively related to BC tumor size and histological grade, as well as positively related to survival probability of BC patients. Uncontrolled abnormal cell proliferation is the foundation of BC development [44]. Besides, cancer recrudescence and metastasis are mainly responsible for BC-related death [4]. The lungs, pleura, bones, skin and soft tissues, liver, and brain are the common metastatic sites of BC [4]. We discovered that LINC00092 overexpression reduced BC MCF-7 and MDA-MB-468 cell proliferation, migration, and invasion. Silence of LINC00092 had contrary influence. Furthermore, LINC00092 overexpression inhibited BC growth *in vivo*. These findings proposed that the lowly expression of LINC00092 contributed to BC progression and implied that LINC00092 is a possible potential biomarker for BC diagnosis and target for BC treatment.

RETRACTED

FLI1 is a key member of the E26 transformation-specific (ETS) family, which is a group of highly conserved transcription factors with a unique winged helix-turn-helix DNA-binding domain [45]. As a pivotal regulator of embryonic development, loss of FLI1 will cause embryonic death [46]. According to the results of pervious literatures, there was controversy about the role of FLI1 in BC development. Scheiber et al. [47] reported that the lower expression of FLI1 in BC meant shorter survival time and stronger degree of malignancy. However, Song et al. [48] discovered that FLI1 was highly expressed in BC tissues, in which expression was positively related to BC progression. Besides, Yan *et al.* [49] also revealed that FLI1 was overexpressed in triple-negative BC subtype and predicted the poor prognosis of BC patients. In the current research, we discovered that FLI1 bound to LINC00092 promoter to positively modulate the LINC00092 expression in BC cells. Similar to LINC00092, FLI1 was also lowly expressed in BC tissues. These findings proposed that low expression of FLI1 at least in part resulted in the low expression of LINC00092 in BC.

As the main manner for BC cells to produce ATP, glycolysis is essential for BC growth [20]. Earlier literature reported that even in aerobic environment, BC cells still will choose glycolysis as the main manner for energy supplement [50]. Chen *et al.* [23] discovered that LINC00092 suppressed cardiac fibroblast activation by regulating glycolysis through an extracellular regulated protein kinase- (ERK-) dependent manner. Zhao et al. [13] revealed that LINC00092 was highly expressed in ovarian cancer cells, which accelerated glycolysis of ovarian cancer cells. However, in this study, we found that silence of LINC00092 accelerated the glycolysis of BC cells via raising glucose consumption and lactate production. LINC00092 overexpression had opposite influence. What is more, inhibition of glycolysis by 2-DG relieved the LINC00092 silence-caused increase of BC cell proliferation. These findings proposed that LINC00092 modulated BC cell proliferation at least via glycolysis. Moreover, these discoveries revealed that LINC00092 might exert distinct regulatory effects on glycolysis in different cancers.

RETRACTED

The imbalance between reactive species and antioxidant defenses will result in the increase of oxidative stress. Excessive amounts of reactive species are detrimental to normal cells, whereas in cancer cells, they lead to accelerated growth and survival related to aggressive and therapy-resistant phenotypes [25]. Mullarky and Cantley [26] discovered that ROS can regulate multiple glycolytic enzymes, including glyceraldehyde 3-phosphate dehydrogenase, pyruvate kinase M2, and phosphofructokinase-1. Martinez-Outschoorn *et al*. [51] found that the mutation of breast cancer susceptibility gene 1 (BRCA1), a key tumor suppressor gene, accelerated oxidative stress and glycolysis in tumor microenvironment of breast cancer. Herein, we also discovered that both glycolysis and response to oxidative stress were modulated by LINC00092 in BC tissues. LINC00092 overexpression reduced the oxidative stress via raising SOD level and lowering MDA and ROS levels in BC cells. However, LINC00092 silence had contrary influence, which activated oxidative stress. These findings proposed that LINC00092 also took part in the modulation of oxidative stress in BC.

The AKT/mTOR pathway is very important for regulation of cell proliferation that is overactivated in many human cancers, including BC, and contributes to neoplastic transformation [39]. More importantly, in recent years, the AKT/mTOR pathway is demonstrated to take part in the regulation of cell oxidative stress and glycolysis [52, 53]. Jia et al. [54] revealed that inhibition of the AKT/mTOR pathway suppressed BC progression through limiting BC cell glycolysis. Zong *et al.* [55] reported that salt-inducible kinase (SIK2), a member of adenosine monophosphate- (AMP-) activated protein kinase family, was beneficial for cisplatin resistance caused by aerobic glycolysis in BC cells via modulating the AKT/mTOR pathway. In recent years, many lncRNAs are discovered to modulate the AKT/mTOR pathway in BC cells [56, 57]. Until now, it is still unclear whether LINC00092 regulates the AKT/mTOR pathway in cells. Herein, we found that LINC00092 silence activated the AKT/mTOR pathway in BC cells, while LINC00092 overexpression had contrary effect. Moreover, activation of the AKT/mTOR pathway by SC79 reversed the LINC00092 overexpression-resulted decreases of BC cell proliferation, migration, invasion, and glycolysis. Inhibition of the AKT/mTOR pathway by MK2206 had opposite influence. These findings proposed that LINC00092 influenced BC cell proliferation, migration, invasion, and glycolysis which could be achieved via the AKT/mTOR pathway.

RETRACTED

For cancer cells, elevated glycolysis alone is not enough to provide all necessary metabolic intermediates for growth and metastasis, and it is also necessary to promote the biosynthesis of the precursor molecules of tricarboxylic acid cycle (TCA) for replenishment [58]. Oxaloacetate is a main precursor molecule of TCA. As a mitochondrial enzyme, PC is responsible for conversion of pyruvate to oxaloacetate in cells [59]. Numerous literatures reported that PC was highly expressed in BC and its high expression was positively related to BC clinical progression, such as tumor size, tumor stage, and poor prognosis [60, 61]. Moreover, PC was discovered to promote BC metastasis [59, 62]. Liu et al. [63] reported that PC could activate the AKT/mTOR pathway in thyroid cancer cells. In the last few years, some literatures have reported the regulatory role of lncRNAs in PC expression in cancer cells [64, 65]. In this research, we revealed that LINC00092 bound to PC to modulate the ubiquitination degradation of PC protein in BC cells. More importantly, overexpression of PC weakened the influences of LINC00092 overexpression on BC cell proliferation, migration, invasion, glycolysis, and the AKT/mTOR pathway. Silence of PC had similar mitigatory activity on the influence of LINC00092 silence on BC cells. These findings proposed that the regulatory function of LINC00092 on PC contributed to the modulatory effects of LINC00092 on BC growth and metastasis.

In general, one lncRNA participates in regulating expressions of multiple proteins and other ncRNAs in cells [11]. As a type of ncRNAs with 18-24 nucleotides, microRNAs are main downstream targets of lncRNA [66]. Zhao et al. [43] reported that LINC00092 sponged microRNA-1827 in BIDC cells to modulate BIDC malignant progression, which implied that LINC00092 regulated BC progression not only by modulating PC expression but also via regulating other molecules. Besides, the *in vivo* experiment in our research was relatively simple. We did not explore the effect of LINC00092 on glycolysis, PC expression, oxidative stress, and the AKT/mTOR pathway *in vivo*. More investigations are still demanded in the future.

Taken together, this research affirmed the tumor-suppressive role of LINC00092 in BC. The low expression of LINC0092 promoted BC cell proliferation, migration, invasion, and glycolysis via the PC-mediated AKT/mTOR pathway. This study revealed that LINC00092 might be regarded as a novel prognostic indicator and potential therapeutic target for patients with BC.

## Figures and Tables

**Figure 1:** LINC00092 was modulated by FLI1 in BC cells. (a, b) Bioinformatics analysis was utilized to predict the relationship between FLI1 and LINC00092. (c, d) Following mock or FLI1 transfection, the FLI1 and LINC00092 expressions in cells were measured via qPCR. *N* = 3. (e, f) ChIP assay was carried out to test the binding between FLI1 and LINC00092 promoter in cells. *N* = 3. (g, h) Dual-luciferase activity assay was carried out to confirm the binding between FLI1 and LINC00092 promoter. *N* = 3. ^N.S.^*P* > 0.05, ^∗^*P* < 0.05, and ^∗∗∗^*P* < 0.001.

RETRACTED

**Figure 2:** LINC00092 regulated BC cell proliferation, migration, and invasion. Following LINC00092 or sh-LINC00092 transfection, the LINC00092 expression in cells (a), cell viabilities (b), proliferation (c), migration (d), and invasion (e) were measured via qPCR, CCK-8 assay, colony formation assay, cell scratch assay, and two-chamber transwell assay, respectively. *N* = 3. ^∗^*P* < 0.05, ^∗∗^*P* < 0.01, and ^∗∗∗^*P* < 0.001.

**Figure 3:** LINC00092 overexpression inhibited BC growth *in vivo*. *In vivo* BC mouse model was established with mock or LINC00092 transfection. (a, b) Body weights and tumor volumes of mice in the mock and LINC00092 group were measured at day 3, day 7, day 14, day 21, and day 28. (c) The visual picture of mice with subcutaneous BC transplantation. (d) The visual picture of tumor tissues and tumor weights was detected. (e) HE staining was carried out to observe the microstructure changes of tumor tissues, and IHC assay was utilized to detect the Ki-67 expression in tumor tissues. *N* = 6. ^N.S.^*P* > 0.05; ^∗∗∗^*P* < 0.001.

**Figure 4:** LINC00092 influenced BC cell glycolysis and oxidative response. (a) GSEA was carried out to explore the enrichment of glycolysis and response to oxidative stress regulated by LINC00092 in BC tissues. (b, c) Following LINC00092 or sh-LINC00092 transfection, cell lactate production and glucose consumption were tested via lactate assay kit and glucose assay kit. *N* = 3. (d, e) Following sh-LINC00092 transfection and/or 2-DG treatment, cell viabilities and proliferation were detected via CCK-8 assay and colony formation assay. *N* = 3. (f) Following LINC00092 or sh-LINC00092 transfection, the SOD, MDA, and ROS levels in cells were tested, respectively. *N* = 3. ^∗^*P* < 0.05, ^∗∗^*P* < 0.01, and ^∗∗∗^*P* < 0.001.

**Figure 5:** LINC00092 influenced BC cell functions and glycolysis via modulating the AKT/mTOR pathway. (a) After LINC00092 or sh-LINC00092 transfection, the AKT, p-AKT, mTOR, p-mTOR, and p-p70S6K protein levels in cells were evaluated by western blotting. *N* = 3. (b) IHC assay was utilized to test p-mTOR and p-P70S6K expressions in mouse xenograft BC tissues. *N* = 6. Following LINC00092 transfection and SC79 treatment, cell viabilities (c), proliferation (d), migration (e), and invasion (f) were tested via CCK-8 assay, colony formation assay, cell scratch assay, and two-chamber transwell assay, respectively. (g, h) Cell lactate production and glucose consumption were tested. *N* = 3. ^∗^*P* < 0.05, ^∗∗^*P* < 0.01, and ^∗∗∗^*P* < 0.001.

RETRACTED

**Figure 6:** LINC00092 regulated ubiquitination degradation of PC protein in BC cells. (a, b) RNA pull-down assay and MS analysis were carried out to identify proteins interacting with LINC00092 in BC cells. *N* = 3. (c) RNA-FISH assay was performed to measure the location of LINC00092 and PC in cells. *N* = 3. (d) The samples from RNA pull-down assay were subjected to western blotting to test PC protein expression. *N* = 3. (e) RIP assay was used to confirm the binding of LINC00092 and PC. *N* = 3. (f, g) Following LINC00092 and sh-LINC00092 transfection, the mRNA and protein levels of PC were tested via qPCR and western blotting. *N* = 3. (h) IHC assay was utilized to test PC expression in subcutaneous BC tissues of mice. *N* = 6. (i) Following LINC00092 (or sh-LINC00092) transfection and CHX treatment, the PC protein level was tested via western blotting in 0, 2, 4, 8, and 12 h. *N* = 3. (j) *In vivo* ubiquitination assay was carried out to test whether LINC00092 modulate degradation of PC protein via the ubiquitination pathway. *N* = 3. ^n.s.^*P* > 0.05, ^∗^*P* < 0.05, ^∗∗^*P* < 0.01, and ^∗∗∗^*P* < 0.001 vs. the mock group; ^#^*P* < 0.05 and ^##^*P* < 0.01 vs. the sh-NC group.

**Figure 7:** Overexpression of PC weakened the influences of LINC00092 transfection on BC cell functions. Following LINC00092 and PC transfection, (a) PC protein levels were tested via western blotting. Cell viabilities (b), proliferation (c), migration (d), and invasion (e) were tested via CCK-8 assay, colony formation assay, cell scratch assay, and two-chamber transwell assay, respectively. (f, g) Cell lactate production and glucose consumption were tested. *N* = 3. ^#^*P* < 0.05, ^##^*P* < 0.01, and ^###^*P* < 0.001*vs.* the mock group; ^∗^*P* < 0.05, ^∗∗^*P* < 0.01, and ^∗∗∗^*P* < 0.001 vs. the LINC00092 group. ^$^*P* < 0.05, ^$$^*P* < 0.01, and ^$$$^*P* < 0.001*vs.* the PC group.

**Table 1:** The primer information for qPCR assay.

Name	Sequence (5′-3′)
LINC00092 forward	AACCAGGAACCTCCGCACCAA
LINC00092 reverse	GCAAGGCTTCCGCAGCTCAA
FLI1 forward	CTACCATGCCCACCAGCAGAAG
FLI1 reverse	CCAGTATTGTGATGCGGCTCCA
PC forward	GCGACGGCGAGGAGATAGT
PC reverse	CCCATGGACTGTTCGGAACTT
GAPDH forward	AAGTATGACAACAGCCTCAAG
GAPDH reverse	TCCACGATACCAAAGTTGTC

## Data Availability

The data used to support the findings of this study are included within the article.

RETRACTED

## Supplementary Materials

Supplementary Materials Supplemental Figure 1: LINC00092 was lowly expressed in BC and negatively related to BC progression. Supplemental Figure 2: FLI1 had lower expression in BC tissues. Supplemental Figure 3: inhibition of the MAPK/mTOR pathway reversed the influence of sh-LINC00092 on BC cell functions and glycolysis. Supplemental Figure 4: inhibition of PC reversed the influence of sh-LINC00092 on BC cell functions and glycolysis. Supplemental Figure 5: PC was involved in the modulation of LINC00092 on AKT/mTOR pathway in BC cells.
